This article has been retracted.

# Screening Tumor-Related Genes of Gallbladder Cancer Based on AR-Based Tumor Expression Profile Gene Chip

**DOI:** 10.1155/2022/8579279

**Published:** 2022-09-26

**Authors:** Jia Guo, Tuotuo Gong, Beina Hui, Xu Zhao, Jing Li

**Affiliations:** Department of Radiation Oncology, The First Affiliated Hospital of Xi'an Jiaotong University, Xi'an 710061, Shaanxi, China

## Abstract

The rapid development of molecular biology and gene chip technology has produced a large amount of gene expression profile data. The main research in this article is to screen the tumor-related genes of gallbladder cancer based on AR-based tumor expression profile gene chip. First, convert the chip data into an expression matrix pattern that can be analyzed, and then standardize and normalize all the data. Run ReliefF, GA, and IReliefF-GA on the data set, record the size of the feature subset, and use the tenfold cross-validation method to obtain the classification accuracy, specificity, and sensitivity of each method on the classifier. The target genes used in the chip were amplified by PCR with the universal primers used in cDNA library construction, and the quality of PCR was monitored by agarose gel electrophoresis. The gene chip data of gallbladder cancer was processed with missing values, singular values, and so forth, and 22294 transcripts were obtained. After statistical testing, there were 9483 transcripts with statistically significant differences. The results show that as the number of clusters increases, the network can be better reconstructed through decomposition modeling.

## 1. Introduction

In recent years, the incidence of cancer has increased year by year, and gallbladder cancer has received more and more attention because of its late detection and higher mortality. Gallbladder cancer ranks fifth to sixth among digestive tract tumors, accounting for 0.1% and 1.1% of general surgical diseases in the same period. The total five-year survival rate is less than 5% due to clinical characteristics such as metastasis to other organs and unresectable tumors. Early diagnosis is the key to a good prognosis. Gallbladder cancer data mining is to systematically mine the prescription experience of clinical diagnosis and treatment of gallbladder cancer and further use the K-means cluster analysis method for analysis and research, so as to make up for the lack of internal and external correlation. Data mining uses database technology to extract the unobvious, undetected, and hidden information and knowledge from the data. It is one of the most popular techniques in data analysis. At present, data mining is widely used in telecommunications, websites, environment, finance, medicine, and other fields.

The analysis of tumor gene expression profile data has important practical significance in clinical treatment. The gallbladder cancer-related genome was screened by expression profiling chip, and the related genes screened by the expression profiling chip were classified and analyzed by bioinformatics, and the exons were selected for PCR amplification and sequencing to clarify the mutation status, in order to develop cDNA chips and gene mutation detection chips related to gallbladder cancer, improve the level of early diagnosis of biliary tract tumors, and provide first-hand information and materials for drugs and gene therapy. The tumor gene expression profile data of tumor patients can be obtained through DNA chip technology, and further analysis can be performed to obtain the early diagnosis results of the diseased tissue, and targeted treatment can be effectively prevented from further deterioration of the tumor. The incidence of gallbladder cancer has been increasing gradually over the years, so it has positive practical significance to study the characteristics of occurrence, development, and metastasis of gallbladder cancer.

AR technology can promote the screening of gallbladder cancer tumor-related genes by tumor expression profile gene chip. C-H uses mRNA data set GSE59102 and miRNA data set GSE70289. After pretreatment, the differentially expressed genes at different tumor stages were selected according to the limma software package. Then, ClueGO was used to perform enrichment analysis on Affymetrix GeneChip protocol to analyze tumor miRNA expression, and Genehese DEGs were used. Based on the BioGRID database, a protein-protein interaction (PPI) network analysis was conducted. Although the mentioned research method is more detailed, it lacks necessary experimental data [1]. Sass et al. determined the growth rate of the tumor by measuring it in two of the latest preoperative MRI scans. They used Affymetrix microarray protocol to analyze tumor miRNA expression and generated CEL files using GeneChip command console software and standardized them using Partek Genomics Suite 6.5. They used statistical software program R to analyze CEL files. They found that tumor miRNA expression was associated with the growth rate of sporadic vestibular schwannomas. Although their experimental method is very comprehensive, it lacks specific research data [2]. Chernaya et al. used real-time RT-PCR to evaluate the expression level of the gene under study. They used allele-specific amplification to determine the BRAF V600E mutation. In addition, they assessed the changes in the expression levels of integrin and osteopontin in benign and malignant tumors. Although their research content is innovative, there are still many loopholes [3]. To identify the networks and pathways of tumorigenesis, Dai used ingenious pathway analysis to identify differentially expressed miRNAs in tumor tissues. Although their research content has a certain reference, it is not precise enough [4]. However, the previously mentioned studies did not use the tumor expression profile gene chip to conduct experiments and research on the tumor-related genes of gallbladder cancer.

By analyzing the gene expression of tumor sample tissues, extract genes that are important to tumors, and establish an effective tumor prediction model. Search for gene changes related to the development of gallbladder cancer, lymph node metastasis, and liver metastasis in the whole genome, so as to know the expression and structural changes of the entire genome, explore the mechanism of gallbladder cancer at the molecular level, and further use molecular biology and molecular pathology methods expanded cases to verify the differentially expressed genes related to gallbladder cancer and lymph node metastasis, making the conclusion convincing.

## 2. Tumor Expression Profile Gene Chip

### 2.1. Data Mining Method of Tumor Expression Profile

These data come from different studies, the research objects may be the same disease, or even the same detection platform is used; therefore, these data have the conditions for integrated analysis. The data mining process mainly includes four processes: data collection, data preprocessing, model establishment, and overall analysis. The integration of multiple data sets can expand the sample size of the research and meet the multicentered sample source, thereby further improving the reliability of the research. With the development of bioinformatics based on computer technology, data integration becomes possible and helps us obtain important biological information from the massive gene expression profile data [5]. The error of expression profile gene chip can be divided into biological error and experimental system error. Biological error mainly refers to sample differences; that is, the expression of specific genes in cells taken from the same tissue is not the same. For biological differences, it is best to perform large replicate experiments. The distance between the sample to be tested and the remaining samples is defined as

(1) $$\begin{array}{c} d\left(X_{i},X_{j}\right)=\sqrt{\sum_{l=1}^{n}{\left(X_{l}^{i}-X_{l}^{j}\right)}^{2}.} \end{array}$$

Usually, due to the independence of the control sample and the experimental data, gene centering can eliminate the influence of the expression value of the control sample by adjusting the value of each gene, such as the mean or median value. Similarly, sample centering can remove certain types of deviations, such as the influence of genes in different spatial positions and background differences on the chip [6]. Another more commonly used standardization process is in the following formula:

(2) $$\begin{array}{c} x_{i,j}=\frac{x_{i,j}-{\bar{x}}_{i}}{\sqrt{1/n-1\sum_{j=1}^{n}{\left(x_{i,j}-{\bar{x}}_{i}\right)}^{2}}}. \end{array}$$

In the above formula, ${\bar{x}}_{i}$ is the average value of the *i*th experiment in the gene expression matrix. If all data are required to be distributed in the range of [0, 1], the following transformation is required:

(3) $$\begin{array}{c} x_{i,j}=\frac{x_{i,j}-\min\left[x_{1,2,\ldots ,n,j}\right]}{\max\left[x_{1,2,\ldots ,n,j}\right]-\min\left[x_{1,2,\ldots ,n,j}\right]}. \end{array}$$

The Lagrange function is as follows:

(4) $$\begin{array}{c} \underset{w,b}{\min}\underset{a}{\max}L\left(w,b,a\right)=\frac{1}{2}{\left\|w\right\|}^{2}-\sum_{i=1}^{n}a_{i}\left[y_{i}\left(wx_{i}+b\right)-1\right], \end{array}$$

where *a*_*i*_(*a*_*i*_ ≥ 0) is the Lagrangian coefficient. The optimal discriminant function is as follows:

(5) $$\begin{array}{c} d\left(x\right)=\mathrm{sgn}\left\{\sum_{i=1}^{l}y_{i}a_{i}^{*}x_{i}x+b_{0}\right\}. \end{array}$$

In the above formula, *y*_*i*_ represents the class label of the support vector *x*_*i*_.

In feature selection, the expression of correlation is as follows:

(6) $$\begin{array}{c} \min R\left(S,C\right),R=\frac{1}{{\left|S\right|}^{2}}\sum_{x_{i},x_{j}\in S}I\left(x_{i};x_{j}\right). \end{array}$$

In the above formula, *R* represents the size of MI between features, and *I*(*x*_*i*_; *x*_*j*_) represents the MI between feature *i* and feature *j*. It can achieve a higher classification accuracy, but it is time-consuming to calculate. Therefore, when the dimension of the original feature set is large, implementing feature selection through Wrapper will make the algorithm more complex [7]. There are many interference factors in the data of gene expression profiling, so there may be errors in the results of expression profiling chip data, and the verification of its reliability is very important.

Due to the characteristics of few samples and high dimensionality of tumor gene expression profile data, feature selection must be performed to reduce the dimensionality in the process of tumor classification feature selection, so as to find genes that have a decisive or important impact on the sample category.

(7) $$\begin{array}{c} C\text{class}=\sum_{j=1}^{n_{g}}\frac{\left|x_{i}-h_{j}\left(x\right)\right|}{\max\left(x\right)-\min\left(x\right)}. \end{array}$$

The characteristic differences between *m*_*j*_(*x*) and *x*_*i*_ are

(8) $$\begin{array}{c} D\text{class}=\sum \frac{p\left(k\right)}{1-p\left(x_{i}\right)}\cdot \sum_{j=1}^{n_{g}}\frac{\left|x_{i}-m_{j}\left(x\right)\right|}{\max\left(x\right)-\min\left(x\right)},i=1,2,\text{…},M. \end{array}$$

First define the mean ${\bar{A}}_{i}$ of all kinds of samples and the overall sample mean $\bar{A}$.

(9) $$\begin{array}{c} {\bar{A}}_{i}=\frac{1}{n_{i}}\sum_{j=1}^{n_{i}}x_{j}^{i},i=1,2,\ldots k,\\ \bar{A}=\frac{1}{n}\sum_{j=1}^{n}x_{j}. \end{array}$$

In the above formula, *x*_*j*_^*i*^ represents the *j*-th sample of the *i*th category. Then calculate the interclass dispersion matrix *S*_*B*_ and the intraclass dispersion matrix *S*_*w*_ of the samples, respectively.

(10) $$\begin{array}{c} S_{B}=\sum_{i=1}^{k}\frac{n_{i}}{n}\left({\bar{A}}_{i}-\bar{A}\right){\left({\bar{A}}_{i}-\bar{A}\right)}^{T},\\ S_{w}=\sum_{i=1}^{k}\frac{1}{n}\sum_{j=1}^{n_{i}}\left(x_{j}^{i}-{\bar{A}}_{i}\right){\left(x_{j}^{i}-{\bar{A}}_{i}\right)}^{T}. \end{array}$$

The expression of the area search space range is as follows:

(11) $$\begin{array}{c} xr_{i}\left(t\right)=\left[xr_{i1}\left(t\right),xr_{i2}\left(t\right),\ldots ,xr_{in}\left(t\right)\right],\;i=1,2,\ldots ,N. \end{array}$$

The formula for determining the regional extreme value is

(12) $$\begin{array}{c} X_{\text{id}}^{rb}\left(t+1\right)=\left\{\begin{array}{c} x_{\text{id}}\left(t+1\right),F\left(x_{\text{id}}\left(t+1\right)\right)<F\left(X_{\text{id}}^{rb}\left(t\right)\right)\\ X_{id}^{rb}\left(t\right),F\left(x_{\text{id}}\left(t+1\right)\right)\geq F\left(X_{\text{id}}^{rb}\left(t\right)\right) \end{array}\right.. \end{array}$$

In the above formula, *X*_id_^*rb*^(*t*) represents the optimal value of the area where the particle is located in the *t*th iteration. Using gene expression profiling data, the expression patterns of genes related to tumor growth at various stages of tumor cell growth can be obtained at any time, providing a basis for tumor diagnosis, treatment, and basic research.

### 2.2. Gene Chip

Gene chip refers to immobilizing a large number of probe molecules (usually higher than 400 per square centimeter) on the support and then hybridizing them with the labeled sample molecules and obtaining the sample molecules by detecting the hybridization signal intensity of each probe molecule. Quantity and sequence information [8]: DNA chip can detect the difference of gene expression between tumor tissue and normal tissue, simultaneously study multiple related parameters from the perspective of disease and drug, and obtain relevant gene function, molecular network, and other information. The integrated analysis technology adopted by the chip has the advantages of high throughput, low consumption, and automation, which is greatly advantageous for tumor biology research [9, 10]. Through the comparative analysis of a large number of differentially expressed genes between gallbladder cancer and normal gallbladder tissues, many new differentially expressed sequences were found, which provided new ideas and clues for the diagnosis and treatment of gallbladder cancer. On the one hand, the gene expression experiment of DNA chip is quite complex, and the objective factors such as instruments and equipment and human factors will have a certain impact on the experimental results, resulting in noise and abnormal values of gene expression profile data. On the other hand, in the process of data processing, there may be errors or sample class marking errors. Through that, the expression levels of thousands of genes can be observed at the same time, so that the life phenomenon and its essence can be studied with a systematic and global concept at the genome level. Therefore, it is necessary to remove irrelevant genes and redundant genes from the original gene set before analyzing gene expression profile data [11, 12]. Although the chip data has certain repeatability, it can only be used as a qualitative or semiquantitative analysis method, not quantitative, and there are certain systematic errors.

In the gene chip experiment, due to the objective influence of some external environment, or sometimes influence by human factors during the experiment, at the same time, the proportion of the real tumor-related features in the data is very small, and there are a large number of tumor-independent features or redundant features will reduce the classification efficiency [13]. Therefore, before classification, we must preprocess the gene expression profile data to remove these interference factors. There is no template for the synthesis of sugar chain; there are only a series of sugar related genes located in an orderly manner. The difference in the expression of sugar related genes will directly lead to changes in the structure of sugar chain [14, 15]. There is a large amount of noisy data and outliers among thousands of features of gene expression profiling data, which will greatly affect our classification accuracy. Gene chip can help comprehensively understand the changes in the genome during the carcinogenesis of the gallbladder. Screening of gallbladder cancer-related genes will help to understand the etiology of gallbladder cancer from the molecular level, find ideal gallbladder cancer markers, and explore the targets of gene therapy. Diagnosis and data of gallbladder cancer have very practical significance.

### 2.3. Gallbladder Cancer Tumor

As we all know, gallbladder cancer is a very aggressive malignant tumor that can metastasize early and cause rapid death. Gallbladder cancer is more common in the neck at the bottom, followed by less in the body. Histologically, adenocarcinoma accounts for 80%, undifferentiated carcinoma accounts for 6%, squamous cell carcinoma accounts for 3%, and mixed carcinoma accounts for 1%. Gallbladder cancer can directly infiltrate the surrounding organs and can also be metastasized through lymphatic blood circulation, nerve bile ducts, and other ways, as well as intraperitoneal implantation, and distant metastasis may occur in advanced patients. Gallbladder cancer spreads through lymphatic metastasis and blood metastasis in the early stage and can directly invade the liver; after the tumor overflows, it can be planted on the surface of the peritoneum, as well as biopsy channels, abdominal trauma, and intraperitoneal implantation. Tumor suppressor genes are genes expressed by normal cells. They can induce cell differentiation, maintain a stable cell state, induce programmed cell death, and regulate cell growth [16, 17].

Once the tumor suppressor gene is inactivated or the activity of its encoded protein is abnormal, it will lead to the uncontrolled cell proliferation and differentiation process, thereby increasing the cell's malignant transformation tendency. The most common causes of gallbladder cancer are gallbladder stones and gallbladder polyps. Repeated stimulation of the gallbladder wall by gallbladder stones can lead to hyperplasia of the gallbladder wall, which is prone to cancerous changes for a long time. Chronic gallbladder inflammation, biliary tract infection, and abnormal biliopancreatic junction are also predisposing factors for gallbladder cancer. Obesity, diabetes, and genetic factors are also high-risk factors for gallbladder cancer. Therefore, for most patients, the accuracy of early imaging and serological examinations of gallbladder cancer means the possibility of patients receiving treatment as soon as possible and also the chance of survival of patients [18]. A vector is a means to introduce an exogenous target gene into the recipient cell and then amplify it in large quantities. The vector itself carries a replicon, so it can replicate and amplify in the host cell with the inserted exogenous target. In addition, the vector also has multiple cloning sites for the insertion of exogenous target gene fragments and also has genetic characteristics such as resistance genes that are helpful for later selection. Generally, the molecular weight of the vector is small, which is suitable for inserting large fragments of foreign target genes [19, 20]. To understand the gene changes in the whole process of carcinogenesis and the dynamic changes of all gene expression in cells in various stages of carcinogenesis, it is necessary to study not just one or a few genes but thousands of genes in the entire genome in various stages from normal to cancerous. There are dynamic changes in gene expression. Similarly, the occurrence and development of gallbladder cancer are the result of the abnormal action of multiple genes and multiple stages.

### 2.4. AR Technology

AR augmented reality is a technology that superimposes virtual data in the real world, providing an interactive window for the experiencer. For application, AR technology uses the computer as the carrier to divide the relevant information into the atmosphere and goals within the scope of virtual space. At the same time, it can return the existing virtual information to the real environment and then organically combine the real space and virtual space. Because its information is the fusion of the real world and the virtual world, the display is more intuitive and convenient for users to make choices and judgments. Virtual reality technology creates a virtual world that completely covers the real world, while augmented reality focuses on the combination of virtual and real worlds. Augmented reality technology depends on the real world, but it will not replace the real world. Instead, it will add its virtual information to the real world to serve the real world. It integrates the real world and the virtual world, extends the virtual world to the real environment through the display, and makes users immerse in the virtual and three-dimensional interactive scene. In general, augmented reality technology complements the real scene but does not completely replace the real scene. Through such virtual reality integration, it provides users with real and virtual dual experience and sensory experience beyond reality, so as to achieve the effect of “enhancement.”

## 3. Tumor Expression Profile Gene Chip Screening of Gallbladder Cancer Tumor-Related Genes Experiment

### 3.1. Experimental Materials

In patients with gallbladder cancer whose intraoperative pathological diagnosis is clear during clinical surgery, gallbladder cancer resection is performed, and gallbladder cancer specimens of different clinical stages and patients' normal gallbladder tissue specimens (gallbladder tissue >5 cm from the edge of gallbladder cancer tissue) will be collected. Good specimens are immediately stored in liquid nitrogen. According to clinical manifestations and pathological diagnosis, as well as clinical grading, Table 1 shows the clinicopathological characteristics of gallbladder cancer patients detected by gene chip.

### 3.2. Chip Data Preprocessing

First, convert the chip data into an expression matrix pattern that can be analyzed, and then standardize and normalize all the data. This experiment is implemented using MATLAB programming, running at 3.40 GHz, a computer with 4 GB of memory, and a 4-core Intel i3-3240 processor and equipped with a 32-bit Windows 7 operating system. Run ReliefF, GA, and IReliefF-GA on the data set, record the size of the feature subset, and use the tenfold cross-validation method to obtain the classification accuracy, specificity, and sensitivity of each method on the classifier. For comparison, the feature size of the original data set and the classification accuracy, specificity, and sensitivity of the original data set on the SVM algorithm are also recorded. The two-dimensional classification problem is a classic machine learning problem. The key is to find a suitable classification plane, and the support vector machine proposes the idea of maximizing the classification distance. Using the methods of visual view analysis, statistical analysis, and biological analysis, through the analysis and comparison of chip data or data comparison between chips, the gene expression in different periods of cell growth, DNA changes in normal tissue and tumor tissue, and DNA before and after medication were determined, as well as changes, genetic mutations, and other complex information.

### 3.3. Chip Hybridization

Gene chip detection of target gene fragments is based on the selective hybridization reaction between probe and target gene nucleic acid. The probe is immobilized on the substrate, and the target gene fragment is loaded onto the chip through the flow channel or sample. The target genes used in the chip were amplified by PCR with the universal primers used in cDNA library construction, and the quality of PCR was monitored by agarose gel electrophoresis. Pathway analysis is performed through online molecular annotation system combined with statistical methods of hypergeometric distribution to preliminarily clarify the biological functions of differentially expressed genes.

### 3.4. Protein Sample Preparation

Complete hybridization means stronger signal, incomplete hybridization means weaker signal, and no hybridization means no signal. Through scanning and detection, combined with the design and distribution information of each point on the chip, various information related to the target gene in the sample can be analyzed and detected. GBD-SD and GBC-SD in logarithmic growth period were selected, respectively. The medium in the culture bottle was gently poured into the waste liquid tank, and then the remaining culture liquid at the bottom of the bottle was sucked up with a pipette, or the remaining culture liquid was sucked up with the absorption effect of absorbent paper. 10 *μ*l PMSF (100 mm) should be added to every 1 ml of pyrolysis liquid and then put on the ice after mixing and shaking.

### 3.5. Screening of Differentially Expressed Genes

All patients' names, gender, age, tumor stage, pathological differentiation, tumor size, growth site, serum CA242, CA125, CA199, and CEA detection values and postoperative survival time were entered into the database.

## 4. Estimation and Analysis of Missing Values in Gene Chip Expression Data

### 4.1. Preselected Gene Set Performance Analysis

In the case of different missing ratios, the curve of the mean value of NRMSE is shown in Figure 1. It can be seen from the figure that the KNN method has the worst effect of all the methods, and KS20 is slightly better than the KNN method. This is because the subsequent SVR in KS20 uses the spatial distribution information between genes; the SVR method has the best effect. For the effect of KS20, KS100, and KS200, this is because the SVR method uses all nonmissing genes to estimate the missing value, while KS20, KS100, and KS200 only use fewer genes, causing a lot of information loss; KS400 is among all the methods in Data 1 and Data 2, KS800 has the best effect. KS800 is the best in Data 3, because an appropriate number of similar genes are selected to estimate the target gene, which not only ensures sufficient information but also excludes irrelevant genes. For interference, it can be seen that, compared with non-time-series data, the estimation accuracies of KNN method and KS20 method in time series data are lower than those of other methods. This means that the missing value estimation of time-series data should adopt an estimation method that can make full use of the correlation information between genes on a sufficient number of training sets.

The number of feature genes and classification performance of various algorithms on different data sets are shown in Table 2. In addition, the serum CA242, CA199, and CA125 levels of gallbladder cancer patients are different from those of GBC patients in clinical stages, and there are significant differences in tumor differentiation and size. The levels of serum CA242, CA199, and CA125 in the gallbladder cancer group were significantly different between the tumor pathological stages IVA, IVB, and II, and they were statistically significant (*P* < 0.05). In the GBC group, the serum levels of the above three tumor markers gradually increased with the progress of tumor clinicopathological stage, tumor size, and differentiation.

The comparison of serum CA242, CA125, CA199, and CEA levels is shown in Table 3. The results show that, with the increase of the number of genes, there is a good positive correlation between the prediction accuracy of the leave one method and the prediction accuracy of the test set, and the change of the prediction curve of the test set is relatively smooth. The clustering results of G data set reflect and verify the fact that all types come from different sources, and the clustering results of a data set also conform to the phenomenon that the characteristics of MLL type cells are very similar to those of AML type and all type cells. The above analysis shows that GA/wv method can be applied to two-class and multiclass classification and can obtain a set of characteristic genes with good generality and reflecting the class structure of samples.

The classification accuracy of different algorithms is shown in Figure 2. It can be seen from the experimental results that the classification accuracy of several classifiers using the sparse representation classification principle is generally higher, which shows that the sparse representation classifier is still suitable for gene expression profile classification, and, according to the classification results of the latter three classifiers, the DPDL dictionary learning algorithm showed the highest classification accuracy on most data sets, and, even on the Colon data set, the classification accuracy of the DPDL algorithm is close to MSRC which has the highest classification accuracy rate. This shows that the algorithm proposed in this paper is effective for gene expression profile data sets. Compared with ordinary sparse representation classification algorithms and dictionary learning classification algorithms, the model in this paper can effectively improve the classification accuracy.

The selection results of different genes are shown in Figure 3. After rearranging the genes with the BW gene selection method, starting from 100 genes to 5000 genes, one gene point was selected for every 100 genes, and finally a total of 50 gene points were selected. The experiment is done with tenfold cross-validation each time, and it runs 20 times each time. We found that only two algorithms, the integrated linear classifier and the integrated *K* nearest neighbors, select the [0, 1] features, and the result of the integrated linear classifier such as the accuracy rate of the positive label reaches 0.992, and the recall rate is 0.984. Compared with the integrated linear classifier, the experimental results of integrated *K* nearest neighbors are not ideal. The experimental results of the simulation data set random forest and integrated support vector machine are not ideal.

### 4.2. Comparative Analysis of Different Classification Algorithms

The classification performance of the core genes in the validation data set is shown in Table 4. The gene chip data of gallbladder cancer was processed with missing values, singular values, and so forth, and 22294 transcripts were obtained. After statistical testing, there are 9483 transcripts with statistically significant differences. After analysis of multiple differences, the differential genes of liver cancer tissues are obtained. High-throughput gene chip data analysis brings a lot of information, and it is difficult to analyze the biological functions of these differential genes.

The effect of NDRG2 expression on GBC-SD cell proliferation is shown in Table 5 and Figure 4. The OD value of GBC-SD-NDRG2 group was lower than that of the blank group (GBC-SD) and that of the control group (GBC-SD-VE) after the three groups of cells were cultured and adherent, and the difference trend became larger and larger with time. The OD values of the two groups were statistically analyzed.

The accuracy of the four feature selection methods for the five data sets is shown in Figure 5. This paper uses the final classifier verification method to evaluate the effectiveness of the feature selection method. The rationality and effectiveness of the feature selection step are measured by comparing the classification performances of different feature selection methods in different data sets. From the perspective of classification accuracy, the SRCMRMR feature selection method proposed in this paper has a generally high accuracy rate and can show very good classification results on different data sets. Especially on the Gliomas data set, compared with other methods, our SRCMRMR method has achieved a great improvement in the classification accuracy. Compared with the MRMR method, the results on other data sets have been significantly improved except for the slightly lower value on the Colon data set, which verifies the effectiveness of this method.

### 4.3. Analysis of the Influence of Genetic Filtering Methods on Experimental Results

The average LOESS curve for all pairwise comparisons of *M* absolute values of nonverified transcripts is shown in Figure 6. The clustering phenomenon of samples in the spatial distribution of comprehensive attributes is obvious, which indicates that, after NMF, the redundant information is eliminated and the category information is highlighted, but a few samples are still not well clustered. The missing value estimation method based on KNN-SVR not only improves the accuracy of missing value estimation but also has high stability, which is helpful for the subsequent analysis to get more accurate results. In Colon dataset, no matter the number of features, the classification accuracy of GSEF algorithm is generally higher than those of other methods, and the average is about 3 percentage points higher; in Lung data set, the classification accuracy of each algorithm is almost the same, and the performance is relatively consistent, because the accuracy of each algorithm is close to 100%, so the improvement effect of GSEF algorithm is not very obvious. On the Lymphama data set, the classification accuracy of GSEF is about 98%, which is higher than those of other methods; similar results can still be found on the prostate data set. It can be seen that the classification accuracy of GSEF algorithm is about 2% higher than those of other methods.

Figure 7 shows the performance comparison results of different projection methods when the training samples are reduced. From the comparison of Figures 7(a) and 7(b), it can be found that, on Leukemia, when there are more than 6 training samples of each type and when the training ratio of each type reaches more than 45% on 11 Tumors, SRC and the algorithm IPRC of this paper have achieved the same performance. Moreover, for the problem of small samples, the accuracy of SRC decreases faster than that of IPRC. When there are only two training samples or the training proportion is only 25%, IPRC is still improved by about 3%. On the colon data set, the average error rates of SRC and IPRC were 13.17% and 11.57%, respectively, which were 1.35% and 1.43% lower than those without gene selection; on the DLBCL dataset, the average error rates of SRC and IPRC were 4.74% and 7.88%, respectively, which were 0.51% and 1.83% lower than those without gene selection. It can be seen that LASSO has better improvement ability than BW for IPRC, so it is feasible to use LASSO for gene selection.

The prediction accuracy rates of the four methods under the KNN and SVM classifiers are shown in Table 6. When the method of randomly dividing the sample set is adopted, the proportion of the training set is 30%, and the proportion of the corresponding test set is 70%, and then the proportion of the training set is increased by 5% until it reaches 70%, and the proportion of the test set is correspondingly reduced by 5%, until it is reduced to 30%. With the increase of the proportion of the training set, the prediction accuracies of PCA, 2DPCA, LDA, and iterative 2DLDA methods also increase correspondingly. The accuracy of the HDM-SVM method when the training data set is less than 50% is higher than those of other classification methods, which shows that, in the classification of data sets with few samples, this method has obvious advantages, and the data set is in after 50%; its accuracy rate is also comparable to other methods, which shows the superiority of the method proposed in this article.

## 5. Conclusions

Accurate classification of tumor data is of great medical significance for the treatment of tumor diseases. These classifications are the summary and generalization of the experience of many pathologists. They divide the various pathological manifestations of a certain disease into many types, which just reflect the disease spectrum of the disease, which can help us systematically recognize and understand how many different performances this disease will have. Through the classification of tumor gene expression profile data, tumor detection can not only predict the tumor type of patients, so as to develop corresponding treatment methods for different patients, but also assist scientific researchers in the development of corresponding tumor drugs. Therefore, the classification and detection of gene expression profile data have very important application value and practical significance. The research on the development of gene expression profile data analysis method will not only improve people's medical science and technology level and improve human health but also promote people's in-depth understanding of biological body and biological process and provide the basis for solving the mystery of life in the future.

With the development of DNA chip technology, a wealth of gene expression profile data has been produced for research and analysis, among which tumor gene expression profile data provides a good source of data for tumor research. Using classification accuracy as a measurement standard, by selecting mainstream classification algorithms for processing tumor data, comparison experiments were carried out on 11 classic data sets, and compared it with the original dataset and the dataset after gene selection. Since various cancers have their gene expression profiles, if the analysis of specific genes at the molecular level can give an accurate diagnosis of cancer, it will have far-reaching significance for the diagnosis and treatment of cancer.

Based on the bioinformatics method, the integration and analysis of gene expression profile data from the public database enable us to further explore the genes that may play an important role in the process of liver cirrhosis progressing into HCC, so as to better reveal the pathogenic process of HCC and open up new ideas. The expression of NDRG2 protein is significantly low in gallbladder carcinoma, and its expression intensity is closely related to the stage, grade, and clinical prognosis of gallbladder carcinoma; NDRG2 protein may play an important role in the development of gallbladder carcinoma from precancerous lesions, and detection of its expression intensity is helpful for early detection of gallbladder carcinoma in precancerous stage. However, the source of the error is brought about by the image acquisition and data analysis process of the chip. The error in this area is related to the scanner, analysis software, and analysis algorithm used, and the related instrument software needs to be improved for reduction.

## Figures and Tables

**Figure 1:** Curve of mean value of NRMSE.

**Figure 2:** Classification accuracy of different algorithms.

**Figure 3:** Selection results of different genes.

**Figure 4:** The effect of NDRG2 expression on the proliferation of GBC-SD cells.

**Figure 5:** The accuracy of the four feature selection methods for five data sets.

**Figure 6:** The average LOESS curve of the absolute value of *M* for all pairwise comparisons of nonchecked transcripts.

**Figure 7:** Performance comparison results of different projection methods when training samples are reduced.

**Table 1:** Clinicopathological characteristics of gallbladder cancer patients detected by gene chip.

No.	Sex	Age	Tum	LN	Dif
1	F	54	T3	N1	MD
2	M	68	T2	N2	WD
3	M	50	T3	N1	MD
4	M	73	T4	N3	PD
5	F	62	T3	N0	PD
6	M	45	T2	N0	PD

**Table 2:** The number of feature genes and classification performance of various algorithms on different data sets.

	Lung		Colon		Leukemia		Prostate	
	Number	Rate	Number	Rate	Number	Rate	Number	Rate
ODP	2880	84.62	2000	81.10	7129	94.44	12600	61.90
SNRS	6	85.44	15	82.26	4	97.36	5	91.18
RF	2880	86.37	2000	84.75	7129	90.18	12600	92.54
SVM	16	86.36	15	84.40	10	94.10	10	90.34
SNRRF	10	89.89	72	87.48	26	94.77	49	93.14

**Table 3:** Comparison of serum CA242, CA125, CA199, and CEA detection levels.

Group	MFI (CEA)	MFI (CA199)	MFI (CA125)	MFI (CA242)
Healthy control group	3.93 ± 2.04	14.97 ± 8.91	10.48 ± 6.38	9.48 ± 3.43
Benign gallbladder disease group	3.83 ± 1.85	15.17 ± 7.82	12.99 ± 6.99	10.19 ± 3.08
Gallbladder cancer group	9.36 ± 3.58	238.17 ± 346.36	55.34 ± 81.78	39.92 ± 45.9

**Table 4:** Classification performance of core genes in the validation data set.

Classification	Sensitivity (%)	Specificity (%)	Accuracy (%)	AUC
Random forest	86.7	82.7	86.8	0.892
Random forest	88.6	85.5	87.6	0.925
SVM	87.8	87.6	87.5	0.923
Decision tree	89.5	90.9	89.4	0.921
Random forest	93.5	91.5	90.6	0.957

**Table 5:** The effect of NDRG2 expression on the proliferation of GBC-SD cells.

Day	GBC-SD	GBC-SD-Ve	GBC-SD-NDRG2	*F* value	*P* value
1	100	100.42 ± 10.73	92.51 ± 6.23	12.66	*P* < 0.01
2	100	99.18 ± 12.54	84.16 ± 7.42	23.78	*P* < 0.01
3	100	101.36 ± 8.41	73.88 ± 10.64	122.53	*P* < 0.01
4	100	102.58 ± 14.59	57.51 ± 9.87	131.66	*P* < 0.01
5	100	100.88 ± 13.62	46.19 ± 3.92	266.51	*P* < 0.01
6	100	98.59 ± 9.27	32.25 ± 7.65	639.16	*P* < 0.01

**Table 6:** The prediction accuracy of the four methods under KNN and SVM classifiers.

Data set	KNN				SVM			
	PCA	2DPCA	LDA	2DLDA	PCA	2DPCA	LDA	2DLDA
ALL	86.79	94.38	94.91	95.32	87.87	93.90	94.89	95.08
DLBCL	55.25	60.54	63.88	66.28	59.17	63.76	63.68	69.38
Lung	90.79	93.20	90.29	93.25	92.23	94.12	90.12	94.15
Novartis	89.06	94.35	93.27	96.38	89.28	94.95	90.68	96.11

## Data Availability

No data were used to support this study.
